This article has been retracted.

# A Study on the Evaluation of the Effect of Exercise on the Treatment of Chronic Diseases Based on a Digital Human Movement Model

**DOI:** 10.1155/2022/1984145

**Published:** 2022-01-31

**Authors:** Yu Meng Guan, Xiao Gui Pan, Ke Chen, Yang Xu

**Affiliations:** College of Physical Education, China West Normal University, NanChong 637000, China

## Abstract

The aim of this study was to summarise the therapeutic effects of exercise interventions for common chronic diseases and to analyse the scope of application and problems of various exercise treatment protocols, with a view to guiding clinical practice and providing references for subsequent research. To this end, this paper describes how to extract feature parameters for gait analysis based on a digital human motion model. In-depth descriptions of the extraction algorithms for spatiotemporal features, centre-of-mass movement features, joint mobility, and joint contact forces are presented, and the reliability of the knee contact force extraction algorithm is analysed in particular. To analyse the effect of exercise on the treatment of chronic diseases, 50 cases of elderly chronic disease patients collected from the community were selected and subjected to healthy exercise for 1 year, before and after the healthy exercise. After the exercise, the elderly chronic disease patients' blood pressure, lipid, and blood glucose attainment rates, chronic diseases, and knowledge of nonpharmacological treatments were significantly higher, with statistically significant differences compared to the preexercise period (*P* < 0.05).

## 1. Introduction

China's health data show that there are more than 300 million patients with chronic diseases (NCD) in China, including about 260 million with hypertension, 100 million with diabetes, 170 million with hyperlipidemia, 110 million with fatty liver, and more than 100 million with overweight or obesity [1]. Health promotion interventions that focus solely on disease treatment or rely solely on the medical and health sector are not effective in promoting the health problems of the Chinese population. Evidence on the value of exercise for the prevention and treatment of chronic diseases is growing, and there is a growing body of evidence on the value of exercise for the prevention and treatment of chronic diseases, and it is possible that, in the near future, sports will become part of medicine. The linkage between sports and medicine will be the most active and cost-effective strategy to prevent and control chronic diseases and maintain the health of the entire population [2]. Also, chronic diseases have become the main cause of death among Chinese residents. The death rate due to chronic diseases is 85%, and the disease burden caused by them accounts for 70% of the total disease burden [3]. Johnston et al. [4] studied the impact of cardiovascular disease on economic growth and found that, for every l% increase in mortality, economic growth in high-income countries fell by 0.1%. Chronic diseases significantly increase healthcare spending, with patients with chronic diseases spending 47.3% more than the average level of healthcare spending.

Exercise has gradually been shown to prevent and treat chronic diseases [5]. Nonpharmacological treatments include moderate exercise.

Exercise is one of the most cost-effective ways to change poor behaviour and lifestyle habits and to prevent and manage chronic diseases. To achieve better results in the prevention and treatment of chronic diseases through exercise, medical exercise professionals need to develop scientific exercise prescriptions that prescribe specific exercise content and volume for the individual patient's physical condition, so as to achieve a scientific and planned preventive fitness or rehabilitation treatment [6].

Exercise prescription refers to a systematic and individualised exercise programme formulated in the form of a prescription given to patients, athletes, and gym-goers by physicians, rehabilitation therapists, and sports instructors according to age, gender, physical health status, and exercise experience, as well as cardiorespiratory functional status and functional level of exercise organs [7]. The exercise prescription should specify frequency, intensity, duration, exercise form, and progression. Recommended aerobic exercise: 3 to 5 d per week at 50% to 80% of exercise tolerance for 20 to 60 min; forms of exercise include walking, treadmill, cycling, rowing, stair climbing, ergometers for the hands and legs, and other appropriate continuous or interval training. Recommended resistance exercise: 2 to 3 d per week, 10 to 15 repetitions per muscle group to achieve moderate fatigue values; forms of exercise include aerobic stretch bands, weight, dumbbells, barbells, pulleys, and weight lifts. Each exercise consists of a warm-up, relaxation, and flexibility exercise. It is recommended to gradually increase the intensity and duration of activity over time and to avoid strenuous physical activity [8].

To this end, this paper describes how to extract feature parameters for gait analysis based on a digital human motion model. The extraction of spatiotemporal features of gait was achieved based on 3D coordinate sequence data of skeletal key points; the subsegmental centre-of-mass weighting method was used to calculate the centre-of-mass movement feature parameters. To analyse the effect of exercise on the treatment of chronic diseases, healthy exercise in the prevention and treatment of chronic diseases can significantly improve patients' clinical indicators and enhance the treatment effect of patients' chronic diseases.

## 2. Related Work

With advances in medical care, the 5-year survival rate for effectively treated cancers has increased significantly and cancer is now classified as a chronic disease [9, 10]. The results in [11, 12] showed that, in the same exercise training population, middle-aged hypertensive patients (41–60 years) had longer-lasting reductions in systolic blood pressure than younger or older patients; women had better blood pressure reduction than men. Regular exercise reduces the risk of hypertension and improves fitness and health. Regular (≥3 days per week) moderate-intensity exercise for a sustained period of time (30–45 min or more) can reduce systolic blood pressure by 5–17 mm Hg and diastolic blood pressure by 2–10 mm Hg [13]. The sustained decrease in blood pressure in hypertensive patients is rapid and pronounced within 24 h after a single exercise session, with a more pronounced trend towards a decrease in systolic blood pressure as the duration of training increases [14].

The results of the US DDD project showed that a lifestyle intervention group that burned 700 kcal/week through at least 7% of body weight found a 58% reduction in the incidence of diabetes in those aged 48–66 years and 71% in those aged ≥60 years after 2.8 years [15]; after 10 years, there was a 34% reduction in the incidence [16]. The combined exercise and diet interventions were effective in controlling the condition of patients with gestational diabetes combined with hyperemesis, balancing indicators of ischaemic and hypoxia damage, and reducing levels of vascular neovascularisation factors, thereby improving maternal and child outcomes in patients [17].

## 3. Digital Human Movement Model

### 3.1. Spatiotemporal Characteristics Required for Gait Assessment

The spatiotemporal parameters used for gait analysis usually include Stride (ST), Step Length (SL) [18], Step Width (SW) [19], Gait Speed (GS) [20], Stride Frequency (SF), Toe Out Angle (TOA), and Support Phase Time Ratio (SPTR). Stance Phase Time Ratio (SPTR) is shown in Figure 1 [21]. The stride length is the distance between the centres of the two ipsilateral feet after one step, expressed in cm. The longitudinal straight-line distance between two points when the right and left heels or toes land successively during walking is called the stride length and is expressed in cm [22]. A step forward with the left foot is called the left stride length, and a step forward with the right foot is called the right stride length. Stride length is significantly related to height; the shorter the stature, the shorter the stride length, with a normal person's stride length being approximately 50–80 cm. The angle of the foot is the angle between the centre line running through the sole of one foot (the long axis of the foot, the line from the midpoint of the heel of the second toe) and the forward direction. The angle of the foot in a normal person is approximately 6.75°.

### 3.2. 3D Coordinate Sequence of Skeletal Key Points

In this paper, we extracted step width, step length, step width, step speed, step frequency, foot deflection angle, and support phase time ratio from the motion trajectory data captured by the Kinect sensor as the spatiotemporal features of gait, and the experimental process is shown in Figure 2. The extraction algorithm can be summarised in the following steps: first, the marker coordinates captured by Kinect are preprocessed to remove coarse errors in the marker coordinates; then, the centre position coordinates of marker points 15 and 16 are calculated to obtain the left plantar coordinates; the centre position coordinates of marker points 19 and 20 are calculated to obtain the right plantar coordinates; then, the Euclidean distance between the unilateral plantar coordinates is used to calculate the average The mean stride width was calculated using the horizontal distance between the left and right plantar coordinates, and the mean stride length was calculated using the distance from the landing of one foot to the landing of the opposite foot; finally, the leg lengths of all subjects were measured; i.e., the Euclidean distances between segments 13–15 and segments 17–19 were calculated, and their mean values were used to normalise stride width, stride length, and stride width. After obtaining the stride length, the stride speed characteristics can be calculated from stride speed = stride length/walking period. The direction of the vector at markers 15 (19) and 16 (20) was used as the direction of the foot deflection angle. In addition, the gait frequency characteristics are calculated by counting the number of steps taken per unit of time; the support phase time is calculated by taking the time when the sole of the foot is in contact with the ground, thus deriving the weight of the support phase time for the complete gait cycle.

### 3.3. Center-of-Mass Movement Characteristics for Gait Analysis

Balance is the ability to maintain the body's stability or the ability to keep the body's centre of gravity within a plane of support. Clinically, balance is the ability of the body to automatically adjust and maintain posture when in a posture or steady state and regardless of position, when moving or when subjected to external forces [23]. It plays an important role in maintaining normal human walking. The centre of gravity is the centre of the body's weight and is the point of action of the combined forces of gravity on the head, torso, and upper limbs. When the body is standing still, the centre of gravity is located between the human sacrum and the umbilicus. When the body is in motion, the centre of gravity changes. The line of gravity is a vertical line drawn through the body's centre of gravity towards the ground. The centre of gravity falls within the plane of support in order for the body to maintain balance. The line of gravity is an auxiliary line for analysing the body's dynamics and can be used to check dynamic patterns and instability. The support surface is the area that supports the body's weight. The area between the bottom of the feet and the area made to contain between the feet when the body is standing is the support surface. When the body is sitting, lying, or moving, the support surface includes the contact surface between the body and the ground and the contact surface between the support surface and the ground, as well as the entire area between the two contact surfaces. The larger the support surface, the more stable the body's centre of gravity and the more balanced the body [24].

The centre-of-mass position of each segment was then calculated using the collected marker positions, and the formula for defining the centre-of-mass position of a body segment is as follows：

(1) $$\begin{array}{c} x_{\text{cm}}=x_{p}l_{p}+x_{d}l_{d};\\ y_{\text{cm}}=y_{p}l_{p}+y_{d}l_{d};\\ z_{\text{cm}}=z_{p}l_{p}+z_{d}l_{d}. \end{array}$$

Finally, the position of the centre of gravity of the body is calculated using the position of the centre of mass of each segment, and the formula is as follows：

(2) $$\begin{array}{c} x_{\text{tcm}}=\frac{\sum_{k=1}^{15}m_{k}x_{k}}{M};\\ y_{\text{tcm}}=\frac{\sum_{k=1}^{15}m_{k}y_{k}}{M};\\ z_{\text{tcm}}=\frac{\sum_{k=1}^{15}m_{k}z_{k}}{M}, \end{array}$$

where *x*_tcm_, *y*_tcm_, and *z*_tcm_ are the coordinates of the body's centre of gravity; *x*_*k*_ and *y*_*k*_ are the coordinates of the *k*th segment; *m*_*k*_ is the mass of the *k*th segment; and *M* is the total mass of the 15 body segments. The range of centre-of-mass movement (up and down and left and right directions) obtained in this paper is shown in Figure 3, on the basis of which the mean values of the range of centre-of-mass movement (L/R distance of COM, L/R COM) and the range of up and down movement (U/D distance of COM, U/D COM) of the subject can be calculated.

### 3.4. Joint Mobility in Gait Analysis

The maintenance of a normal gait involves the participation of the trunk, pelvis, hip, knee and ankle joints, lower limb muscles, and the upper limbs and is a complex and coordinated movement. Walking is also a three-dimensional spatial activity, so gait should be analysed from three perspectives. In the sagittal view, the gait is observed from the side, and eight frames are taken for analysis according to the EFG division of gait, analysing the angles taken by the hip, knee, and ankle joints at different stages. The upper part of the trunk should be upright, with a slight forward lean as the speed increases, and the upper limb should be swinging in the opposite direction to the lower limb movement, which reduces the trunk swing to maintain balance. The shoulder joint swings freely at 32°, flexes at 8°, and extends at 24°. In coronal plane observation, the gait is observed from the front or from behind, and the upward and downward movement of the centre of gravity are analysed as shown in Figure 4.

The specific process is expressed as *L*_1_, *L*_2_, and *L*_3_, respectively. *L*_1_ was calculated as in equation (3), and the rest of the distances were calculated in a similar way. Finally, the knee flexion angle *α* is calculated using the triangle method in motion space, and the formula is shown in equation (4).

(3) $$\begin{array}{c} L_{1}=\sqrt{{\left(X_{\text{hip}}-X_{\text{knee}}\right)}^{2}+{\left(Y_{\text{hip}}-Y_{\text{knee}}\right)}^{2}+{\left(Z_{\text{hip}}-Z_{\text{knee}}\right)}^{2}}, \end{array}$$

(4) $$\begin{array}{c} \alpha =180^{{}^{\circ}}-\arccos\left(\frac{L_{1}^{2}+L_{2}^{2}-L_{3}^{2}}{2\times L_{1}\times L_{2}}\right)\times \frac{180^{{}^{\circ}}}{\pi }. \end{array}$$

The hip flexion and extension angle is measured using the spatial vector method, as shown in Figure 5, in the following way：

(5) $$\begin{array}{c} \overset{⟶}{s_{1}}=\left(X_{hc}-X_{\text{spinal}},Y_{hc}-Y_{\text{spinal}},Z_{hc}-Z_{\text{spinal}}\right). \end{array}$$

The hip-to-knee vector is set to

(6) $$\begin{array}{c} \overset{⟶}{s_{2}}=\left(X_{\text{hip}}-X_{\text{knee}},Y_{\text{hip}}-Y_{\text{knee}},Z_{\text{hip}}-Z_{\text{knee}}\right). \end{array}$$

Let the hip joint flexion angle be *β*, calculated as shown in the following equation:

(7) $$\begin{array}{c} \beta =\arccos\left(\frac{\overset{⟶}{s_{1}}\cdot \overset{⟶}{s_{2}}}{\left|\overset{⟶}{s_{1}}\right|*\left|\overset{⟶}{s_{2}}\right|}\right)*\frac{180^{{}^{\circ}}}{\pi }. \end{array}$$

### 3.5. Joint Contact Forces for Gait Analysis

This paper proposes the use of an RGB-D data-driven bone muscle model to predict knee contact forces during walking, with the potential of Microsoft's RGB-D camera Kinect as a new alternative tool due to its low cost, ease of operation, and low spatial constraints. Validation of its accuracy revealed that the deviation between the results measured by the Qualisys motion capture data-driven bone muscle model and those measured by the RGB-D data-driven bone muscle model ranged from 57.8 to 90.7 N, confirming the ability of the RGB-D data-driven bone muscle model to accurately predict knee contact forces during walking of the subject. The Pearson correlation coefficients for the two measures ranged from 0.943 to 0.988, showing perfect waveform similarity between the two measures. The RGB-D data-driven bone muscle model is, therefore, able to accurately predict knee contact force and could be used as a better alternative in clinical practice, as shown in Figure 6.

## 4. Case Studies

Fifty elderly patients with chronic diseases in the community collected from February 2017 to December 2018 were selected and given healthy exercise for 1 year. All patients met the diagnostic criteria. Among the patients, 26 were male and 24 were female, aged 60 to 87 years, with an average of (74.3 ± 0.5) years. There were 30 cases of hypertension and 20 cases of diabetes mellitus [25].

After the health exercise, the elderly patients with chronic diseases had significantly higher rates of attainment of blood pressure, blood lipid, and blood glucose standards and knowledge of chronic diseases and nonpharmacological treatments, with statistically significant differences compared with those before the exercise (*P* < 0.05), as shown in Table 1.

The change in patients' chronic disease behaviour was significantly higher after the health campaign than before the health campaign, with a statistically significant difference (*P* < 0.05), as shown in Table 2.

## 5. System Effects

Healthy exercise is a comprehensive exercise to control health risk factors of individuals and groups. Healthy exercise is carried out for elderly patients with chronic changes in the community, and special health exercise groups are established to comprehensively assess patients' disease conditions, develop scientific health programmes, and provide targeted and personalised guidance to elderly patients with chronic diseases. In this study, the rate of elderly patients with chronic diseases meeting blood pressure, blood lipid, and blood glucose standards and knowledge of chronic diseases and nonpharmacological treatments increased significantly after the health campaign, with a statistically significant difference compared to the rate before the campaign (*P* < 0.05). After the health campaign, the change in patients' chronic disease behaviour was significantly higher than before the health campaign, with a statistically significant difference (*P* < 0.05), as shown in Figure 7.

It is evident that health campaigns can achieve good results in the management of chronic diseases, improving all clinical indicators and reinforcing the behavioural change profile of patients with chronic diseases. The treatment of chronic respiratory-related diseases (e.g., chronic bronchitis, bronchial asthma, and chronic obstructive pulmonary disease) has been found to reduce patients' healthcare costs by 60% compared to the same period using this integrative model of physical medicine [26]. Weight loss through exercise and other forms of activity that increase energy expenditure can reduce initial body weight by 9–10%, and exercise can prevent weight regain. Exercise did not exacerbate the clinical symptoms or the inflammatory response of children with mild-to-moderate asthma. Extending the duration of exercise combined with increasing the frequency of exercise was the most effective way to reduce body weight, as shown in Figure 8.

Long-term adherence to exercise can be an effective means of preventing the development of osteoporosis in older diabetic patients [27]. Exercise-cognitive interventions can effectively improve cognitive function, enhance daily living skills, and alleviate adverse mood in patients with cognitive impairment[28]. Exercise has a preventive and therapeutic effect on psychological disorders and has a positive effect on developing good psychological quality, promoting mental health, improving mood and state of mind, improving sleep quality, and promoting dopamine secretion, as shown in Figure 9.

We recommend that all patients with chronic diseases should be assessed by clinical professionals before exercising and that exercise plans should be developed to suit individual needs, taking into account the patient's physical condition and that scientific and reasonable individualised exercise prescriptions should be established to bring practical benefits to the health of the nation so that the general public can actively participate in the “Healthy China” which is the trend of the times.

## 6. Conclusions

This paper describes how to extract feature parameters for gait analysis based on a digital human motion model. Algorithms for extracting spatiotemporal and mass movement parameters, joint mobility, and joint contact forces are described in depth, and the reliability of the knee contact force extraction algorithm is analysed in particular. Rationalised exercise prescription can reduce the incidence of malignant tumours and improve the survival and physical performance of patients with malignant tumours, reduce the prevalence of cardiovascular disease and the risk of death, lower blood pressure, improve blood glucose and reduce the use of hypoglycaemic drugs, promote pulmonary rehabilitation, control body weight, and prevent and treat psychological disorders.

## Figures and Tables

**Figure 1:** Schematic diagram of the spatiotemporal characteristics of gait.

**Figure 2:** Schematic diagram of the gait feature extraction experiment.

**Figure 3:** Range of movement of the centre of mass.

**Figure 4:** Calculation of knee flexion and extension angles using the spatial triangle method.

**Figure 5:** Calculation of hip flexion and extension angles using the space vector method. (a) Morphological ACWE segmentation. (b) Morphological ACWE evolution. (c) Morphological GAC segmentation. (d) Morphological GAC evolution.

**Figure 6:** Knee joint contact force distribution curve for the complete gait cycle.

**Figure 7:** Effect of treatment with different exercises.

**Figure 8:** Healing effect of different lengths of exercise.

**Figure 9:** Confusion matrix for postexercise effects.

**Table 1:** Changes in clinical indicators of patients before and after healthy exercise [*n* (%)].

Time	Number of cases	Blood pressure standard	Blood lipid standard	Blood glucose standard	Nondrug treatment awareness	Knowledge of chronic diseases
Before management	50	14	21	18	27	26
After management	50	31	30	36	43	42

**Table 2:** Changes in chronic disease behaviour before and after healthy exercise [*n* (%)].

Time	Number of cases	Quit smoking and alcohol	Low fat and low salt intake	Exercise	Compliance with medical advice	Medication compliance
Before management	50	20	16	12	18	26
After management	50	40	38	41	44	43

## Data Availability

The datasets used during the current study are available from the corresponding author on reasonable request.
